The article "Assessment of patient safety measures in governmental hospitals in Al-Baha, Saudi Arabia" was published in 2019. Journal: AIMS Public Health.

# Assessment of patient safety measures in governmental hospitals in Al-Baha, Saudi Arabia

**DOI:** 10.3934/publichealth.2019.4.396

**Published:** 2019-10-15

**Authors:** Mohamed AwadElkarim Mohamed Ibrahim, Osman Babiker Osman, Waled Amen Mohammed Ahmed

**Affiliations:** 1 Public Health Department, Faculty of Applied Medical Sciences, Albaha University, Saudi Arabia; 2 Nursing Department, Faculty of Applied Medical Sciences, Albaha University, Saudi Arabia

**Keywords:** patient safety, application, Al-Baha, hospital, health care providers

## Abstract

**Background/objective:**

There is a need for patient safety in healthcare settings, WHO recommended an intergradation of patient safety in the curriculum of health specialties. This study aimed to assess the application patient safety measures at governmental hospitals in Al-Baha region.

**Methods:**

This is a descriptive cross-sectional study. It was conducted at Al-Baha governmental hospitals, 2017–2018. The data was collected using a pretested, modified and validated questionnaire, a convenience sampling technique was used among 115 health care providers (doctors and nurses). The collected data was analyzed using SPSS version 22.

**Results:**

The study showed that most of participants have previous training on patient safety and about 81.7% of them had heard about global aims of patient safety. The level of application of patient safety at Al-Baha governmental hospitals was 106 (92.2%) as very often. The findings showed that there are no significant influencing factors on application of patient safety.

**Conclusion:**

The application of patient safety in Al-Baha governmental hospitals was very high. There are no significant influencing factors for the application status of patient safety measures in Al-Baha governmental hospitals.

## 1. Introduction

Patient safety, medical errors and adverse event are a major matters in health care systems across the world [1]. Patient safety is an extensive topic from basic skills and extended to high modern technology and reforming hospitals and services of washing hands correctly and being as a team. Patient safety involves responsibility of individuals to practice safely, health care providers can improve patient safety by targeting patients and their families in examination procedures, educating from mistakes and communicating effectively with the health-care providers [2]. The application of a patient safety measures was recommended earlier by the Institute of Medicine to ensure application of patient safety [3],[4]. The assessment of the application level for safety measures is a corner stone for launching a patient safety culture [5].

The safety of patients is an important indicator of the quality of health care. The continuing development of a high quality health services which depends on evidence-based medicine, which leads to reduce medical errors, 75% of adverse events related to systemic organization but not individual error [6],[7], 50–80% of the errors can be avoided [2],[8]. Researches, by WHO in seven regional countries, (Pakistan, Afghanistan, Sudan, Iraq, Egypt, Morocco and Yemen) showed that among each four individual injections three of them were not reliable, which expose the patients to the danger of abscesses and infection as hepatitis B,C and HIV virus [9]. The previous studies mainly investigated the effects, validity and reliability of patient safety program. Oman is one of the gulf countries that have a national patients safety programs which have been implemented. They also did the first international patients safety conference was held in 2011, in the conference countries such as Sudan, The United Arab Emirate and Qatar viewed their experience concerning their established national patient safety programs, however the establishment of patient safety program by WHO in 2004 was recommended for all members of world health assembly. The situation of patient's safety in most countries is still under consideration According to Saudi Arabian hospitals surveys, there are a need to expand and focus on quality and application of patient safety [10]–[14].

The article "Assessment of patient safety measures in governmental hospitals in Al-Baha, Saudi Arabia" was published in 2019. Journal: AIMS Public Health.

The patient safety is one of the significant dimensions of quality and systematic development of the medical process. In high income countries, reports indicate that adverse events in the operation room represent 48% of all adverse events and 2% of all hospitalized patients and 74% are preventable [15], in addition to the great increase of the need for patient safety measures, as recommended by WHO to integrate patient's safety program in all health specialties curriculum. This study assessed the application level of all aspects of patient safety by healthcare providers which could help health authorities to identify their prevailing drawbacks in field of patient safety [16], and permit the hospitals to measure their application level [17]. The Previous studies in Saudi Arabia have showed that key indicator for measuring patient safety in hospitals include communication, a high quality instructions, common understanding of the importance of patient safety, participation of the hospitals and system for reporting medical error [10]–[14].

Furthermore, previous reports had stated that the culture of patient safety require more investigations, concerning event reporting by the healthcare providers, the hospital plans to applying patient safety measures [10],[18]. However, many previous studies have been conducted to assess on the distribution and patient safety measures, there is no traced reports investigating application of patient safety measures in Saudi Arabia hospitals. Thus, the study was assumed to provide information about the current status of patient safety application at governmental hospitals in Al-Baha. Distributing research findings to international audiences may be useful in terms of learning about research methods and encouraging continued investigations on patient safety in each nation. Moreover, the topic investigated patient safety measures in well stablished hospitals is a cornerstone to initiate the situation. For example, discovering medical errors using the scientific methods with a real interest of researchers from academic and clinical settings makes the urge to engage the international audience.

The article "Assessment of patient safety measures in governmental hospitals in Al-Baha, Saudi Arabia" was published in 2019. Journal: AIMS Public Health.

## 2. Methods

### 2.1. Study design

This is a descriptive cross-sectional hospital-based study. It was conducted in Al-Baha governmental hospitals. The study aimed to assess the application patient safety measures in governmental hospitals in Al-Baha region.

### 2.2. Study place

The study was enrolled in two governmental referral hospitals in Al-Baha region (Aqiq General Hospital and Prince Mashari Hospital), 2017–2018.

### 2.3. Study population

The sample size was calculated using computerized sample calculator (on the software the information was entered as follow: population size = 498, Power = 0.5, confidence level = 95%, and confidence interval = 8, the calculated sample size was 115; the convenience sampling technique was used to collect the data. The frame of healthcare provider (HCPs) was 498 who working the selected hospital, due to time factor the available HCPS were enrolled in this survey. The included HCPs were working in the two hospitals as permanent workers as nurses or doctors. The interns, administrators and other healthcare providers were excluded from this study.

### 2.4. Data collection

The data was collected using questionnaire for demographic data and checklist for application status of patient safety measures by HCPs. The questionnaire was adopted from previous questionnaires on patient safety [19]–[21], then was tested and validated. The Cronbach alpha was above acceptable level. The questionnaire includes two parts; part one for demographic variables of HCPs (Age, experiences, training and occupation), part two consists of 31 items for application of patient safety in the hospitals.

### 2.5. Data management

The collected data was analyzed using the software of Statistical Package for Social Science (SPSS) version 22. The frequency and percentages were represented in tables, charts and graphs; then Chi-square test was performed to test the significance of relationship.

The article "Assessment of patient safety measures in governmental hospitals in Al-Baha, Saudi Arabia" was published in 2019. Journal: AIMS Public Health.

### 2.6. Ethical considerations

Prior to the study, the aim has been explained and clarified by the researchers and participants. A written permission was obtained from ministry of health and hospitals authority before participation in the study. Participants' confidentiality, privacy and dignity were guaranteed. Identity of study subjects was protected. The study was funded by the Deanship for scientific Research at Albaha University who ethically approved the study and sent a letter to Al Baha Health Affairs.

## 3. Results

A total of 115 healthcare providers (HCPs) (doctors and nurses) participated in this study. The demographics characteristics were summarized in Table 1. The age of HCPs were mainly between 20 to 40 years 101(87.8%). The participants in this study were 112 (97.4%) nurses and 3 (2.6%) doctors. They have working experiences less than 5 years 52(45.2%), 5 to 10 years 54(47%) and only 9(7.8%) more than 10 years. Most of participants 91(79.1%) have previous training on patient safety, Table 1 About 81.7% of HCPs had heard about global aims of patient safety, Table 1.

The application of patient safety in Al-Baha governmental hospitals were reported in Table 2. About 106 (92.2%) of HCPs applied very often patient safety measures in the working place and 9(7.8%) of them applied patient safety measures often during their work in the hospitals.

There are many influencing factors for the application status of patient safety measures in Al-Baha governmental hospitals by HCPs. The findings in Table 3 showed that the relationships between the factors (working hospital, HCPs age, job title, previous experiences and previous training in patient safety) and application level are insignificant.

**Table 1.** Demographic characteristics of health care providers in Al-Baha governmental hospitals, Saudi Arabia.

Variable		Frequency (n = 115)	%
Working Hospital	Aqiq General Hospital	26	22.6
	Prince Meshari Hospital	89	77.4
Age	< 20 years	8	7
	20–40 years	101	87.8
	> 40 years	6	5.2
Job title	Doctor	3	2.6
	Nurse	112	97.4
Working Experiences	< 5 years	52	45.2
	5–10 years	54	47
	> 10 years	9	7.8
Training on patients safety	Yes	91	79.1
	No	24	20.9
Hearing of global patient safety goals	Yes	94	81.74
	No	21	18.26

**Table 2.** Health care providers' application for patient safety measures in Al-Baha governmental hospitals, Saudi Arabia.

Application item	Never n (%)	Almost never n (%)	Sometimes n (%)	Fairly often n (%)	Very often n (%)
Correct understanding of patient very shift	0(00)	0(00)	6(5.2)	16(13.9)	93(80.9)
Restrict dealing with dangerous drug.	3(2.6)	2(1.7)	9(7.8)	15(13)	86(74.8)
Good communication style between patient and health care providers.	0(00)	0(00)	3(2.6)	25(21.7)	87(75.7)
Make sure of the concerned patient in case of surgical operations and the correct procedures.	0(00)	3(2.6)	1(0.9)	10(8.7)	101(87.8)
Reduce the risks of hospital infection.	0(00)	0(00)	5(4.3)	15(13)	95(82)
Identification of patient done through his full name.	0(00)	0(00)	0(00)	4(3.5)	111(96.5)
Clearly written of patient instructions is used.	0(00)	0(00)	0(00)	13(11.3)	102(88.7)
Dangerous drugs are prescribed by physician only.	1(0.9)	0(00)	0(00)	12(10.4)	102(88.7)
Review of the drug, doses and time for each drug you want to give.	2(1.7)	0(00)	3(2.6)	7(6.1)	103(89.6)
Sterilizing the site of injection.	4(3.5)	0(00)	1(0.9)	14(12.2)	96(83.5)
Do not remove needle from the used syringes.	2(1.7)	0(00)	2(1.7)	20(17.4)	91(79.1)
Dispose the used syringes and needles in safety boxes.	0(00)	0(00)	2(1.7)	18(15.7)	95(82.6)
Make sure of correct dose.	0(00)	0(00)	4(3.5)	19(16.5)	92(80)
Explain the procedure for patient.	0(00)	1(0.9)	2(1.7)	15(13)	97(84.3)
Wash your hands before dealing with patients.	0(00)	0(00)	3(2.6)	3(2.6)	101(87.8)
Wash your hands after dealing with patients.	1(0.9)	4(3.5)	0(00)	6(5.2)	104(90.4)
Wash your hands after finishing work.	0(00)	2(1.7)	1(0.9)	12(10.4)	100(87)
Wash your hands when touching any suspected material to be contaminated.	0(00)	2(1.7)	1(0.9)	14(12.2)	98(85.2)
My supervisor/manager says a good word when he/she sees a job done according to established correctly.	7(6.1)	7(6.1)	25(21.7)	29(25.2)	47(40.9)
My supervisor/manager seriously considers staff suggestions for improving the care.	8(7)	5(4.3)	24(20.9)	22(19.1)	56(48.7)
After we make changes to improve the health services, we evaluate their effectiveness.	6(5.2)	1(0.9)	25(21.7)	36(31.3)	47(40.9)
Mistakes have led to positive changes here.	16(13.9)	8(7)	6(5.2)	28(24.3)	57(49.6)
We have enough staff to handle the workload.	26(22.6)	6(5.2)	15(13)	25(21.7)	43(37.4)
Healthcare staff receive training in patient safety.	7(6.1)	12(10.4)	14(12.2)	23(20)	59(51.3)
It is very unusual for patients to be given the wrong drug.	5(4.3)	13(11.3)	8(7)	17(14.8)	72(62.6)
The nurses will be committed to identifying and addressing patient safety risks.	1(0.9)	0(00)	9(7.8)	23(20)	82(71.3)
The doctors will be committed to identifying and addressing patient safety risks.	19(16.5)	7(6.1)	10(8.7)	24(20.9)	55(47.8)
The hospital will not criticize me for making mistakes.	5(4.3)	2(1.7)	29(25.2)	22(19.1)	57(49.6)
Managers in the healthcare system will make it easy to report errors.	3(2.6)	4(3.5)	28(24.3)	30(26.1)	50(43.5)
Admitting an error I had made would lead to just and fair treatment by management.	4(3.5)	3(2.6)	22(19.1)	30(26.1)	56(48.7)
I am able to talk about my own errors.	8(7)	0(00)	22(19.1)	27(23.5)	58(50.4)
Overall level of application.	0(0%)	0(0%)	0(0%)	9(7.8%)	106(92.2%)

The article "Assessment of patient safety measures in governmental hospitals in Al-Baha, Saudi Arabia" was published in 2019. Journal: AIMS Public Health.

**Table 3.** Relationship between health care providers influencing factors and overall level of application for patient safety measures in Al-Baha governmental hospitals.

ApplicationHCP criteria		Never n (%)	Almost never n (%)	Sometimes n (%)	Fairly often n (%)	Very often n (%)	*p*-value
Working Hospital	AGH	0(0)	0(0)	0(0)	4(15.4)	22(84.6)	0.1
	PMH	0(0)	0(0)	0(0)	5(5.6)	84(94.4)	
Age	< 20 years	0(0)	0(0)	0(0)	0(0)	8(100)	0.2
	20–40 years	0(0)	0(0)	0(0)	8(7.9)	93(92.1)	
	> 40 years	0(0)	0(0)	0(0)	1(16.7)	5(83.3)	
Job title	Doctor	0(0)	0(0)	0(0)	0(0)	3(100)	0.6
	Nurse	0(0)	0(0)	0(0)	9(8)	103(92)	
Working Experiences	< 5 years	0(0)	0(0)	0(0)	2(3.8)	50(96.2)	0.3
	5–10 years	0(0)	0(0)	0(0)	6(11.1)	48(88.9)	
	> 10 years	0(0)	0(0)	0(0)	1(11.1)	8(88.9)	
Training on patients safety	Yes	0(0)	0(0)	0(0)	8(8.8)	83(91.2)	0.4
	No	0(0)	0(0)	0(0)	1(4.2)	23(95.8)	

*Note: HCP = Health Care Providers; AGH = Aqiq General Hospital; PMH = Prince Meshari Hospital; * = significant.

## 4. Discussion

The level of application of patient safety measures by health care providers at Albaha Governmental hospitals was high. These findings supporting the results of one study conducted in Riyadh, Saudi Arabia which showed increase HCPs attention on patient safety and continuous improvement in this field [11], on the other hand, the finding of recent study conducted in Almadinah Almonawarah, Saudi Arabia which showed that nurses in governmental hospitals have negative attitude and perception towards patient safety culture [10]. A systematic review for measuring patient safety climate showed that all previous surveys covered the five main aspects of patient safety including leadership, policies and procedures, staffing, communication and reporting [19]. Contradicting findings were also reported from many countries; nurses graded their hospitals as poor safety in Switzerland (4%) in Poland (18%) [22].

The HCPs understanding on communication style with their patients was very often as good communication, they mainly identify their patients with full name, and explain procedure for patients. The application of measures on the risk management was investigated which showed that measure to reduce risk of hospital infections was very high concerning restriction of dangerous drugs, sterilization for surgical interventions, washing hand at appropriate times and dealing with wrong doses. that supports the findings by Simsekler which showed a developing agreement between the risk management in healthcare settings that support the application of multiple risk management measures [23]. Furthermore a study conducted by Gurses to identify and categorize patient safety hazards in specific operating rooms which showed that HCPs have non-adherence to applying evidence-based practices [24].

The article "Assessment of patient safety measures in governmental hospitals in Al-Baha, Saudi Arabia" was published in 2019. Journal: AIMS Public Health.

The findings of this study showed that the relationships between the mentioned factors and application of patient safety measures are insignificant. In comparison to other studies on the factors influencing the application of patient safety in hospitals, there are many previous studies were found. A study conducted in Florida, United State showed that the use of information technology has direct positive effect on the application of patient safety [25], another study on the medication safety showed that using a computerized medication ordering improved patient safety in the hospital [26]. On the other hand, an inverse relationship between patient safety and quality of the hospital [27]. In a similar way a study by Simsekler investigated the link between healthcare risk identification and patient safety which showed that patients safety is influenced by inadequate HCPs training, a requirements for financial efficiency and patient safety [28].

The strengths of this study are the study conducted on 115 nurses and doctors, and a very important topic has been studied. The study limitations include; the selected hospitals, which represent a limited geographical area thus reducing its generalizability.

## 5. Conclusion

To sum up, this study showed a high level of application for patient safety measure by HCPs at two governmental hospitals in Al-Baha region, Saudi Arabia. There is insignificant relationship of working area, age of HCPs, job title, previous experiences and previous training with application level. It is recommended to conducted in-depth investigation for the application status of patient safety in all governmental hospitals.
